# Long non-coding RNA MACC1-AS1 promoted pancreatic carcinoma progression through activation of PAX8/NOTCH1 signaling pathway

This article has been retracted.

**DOI:** 10.1186/s13046-019-1332-7

**Published:** 2019-08-07

**Authors:** Chen Qi, Chen Xiaofeng, Li Dongen, Yang Liang, Xu Liping, Hu Yue, Jiang Jianshuai

**Affiliations:** Department of Hepatobiliary & Pancreatic Surgery, Ningbo First Hospital, No. 59 Liuting Street, Haishu District, Ningbo, 315000 Zhejiang Province China

**Keywords:** Pancreatic carcinoma (PC), Long ncRNAs (lncRNAs), Pyruvate kinase M2 (PAX8), Proliferation, Metastasis

## Abstract

**Background:**

Accumulated evidences have demonstrated that long non-coding RNAs (lncRNAs) are dysregulated and correlate with the pathophysiological basis of malignant tumors. The objective of this research is to uncover the possible molecular mechanism of MACC1-AS1 regarding the regulation of pancreatic carcinoma (PC) metastasis.

**Methods:**

lncRNA microarray and qRT-PCR were applied to identify differentially expressed lncRNA profile in PC. The function and role of MACC1-AS1 in PC were assessed via in vitro as well as in vivo assays. Luciferase analyses, RNA immunoprecipitation, and RNA pull-down were performed to determined the underlying MACC1-AS1 mechanisms.

**Results:**

Numbers of differentially expressed lncRNAs in PC were identified via lncRNA microarrays, among which MACC1-AS1 was revealed as the most abundant lncRNA. The upregulation of MACC1-AS1 in PC was further confirmed in two expanded PC cohorts, which showed that MACC1-AS1 expression was upregulated in those PC patients with poor survival. Functionally, knockdown of MACC1-AS1 inhibited the proliferation as well as metastasis of PC cells. Meanwhile, MACC1-AS1 upregulated the expression of PAX8 protein, which promoted aerobic glycolysis and activated NOTCH1 signaling. Additionally, PAX8 was upregulated in PC tissues, which was correlated with the expression of MACC1-AS1 and the overall survival of PC patients.

**Conclusions:**

Together, our findings indicate a critical role of MACC1-AS1/PAX8/NOTCH1 signaling, which may be an alternative treatment target in PC therapy.

**Electronic supplementary material:**

The online version of this article (10.1186/s13046-019-1332-7) contains supplementary material, which is available to authorized users.

## Background

Globally, pancreatic carcinoma (PC) is the fourth leading cause of cancer-related death, which is one of the most aggressive tumors [1, 2]. Currently, complete tumor resection is considered the only potential treatment for PC that results in a complete cure [3]. Normally, the tumor would remain concealed in the early stages, whereas it could progress fast; therefore, the disease of most patients is found during the advanced stage [4]. Recent findings have uncovered that approximately 98% of human genome transcripts are ncRNAs, which have little or even no protein-coding capability [5]. LncRNAs, which are no less than 200 nt in length, are dominant in the ncRNA family [6]. Accumulated investigations have showed that lncRNAs are critically involved in the carcinogenesis and development of carcinomas of human, including PC [7].

Some lncRNAs, including NORAD, PVT1, and CASC2, are reported with aberrant expressions in PC, which can regulate tumorigenesis and progression of PC [8–10]. Nevertheless, the mechanisms and functions of them in PC are poorly known.

In this investigation, by using lncRNA expression microarrays, we found a bunch of lncRNAs aberrantly expressed in PC tissues. Further validation in two PC cohorts revealed that MACC1-AS1 was increased in most of PC tissues, which was involved in PS. Functional studies confirmed that MACC1-AS1 enhanced PC cell metastasis and proliferation. Mechanistic analyses uncovered that MACC1-AS1 promoted carcinogenesis and progression through binding to pyruvate kinase M2 (PAX8) and enhancing the aerobic glycolysis and NOTCH1 signaling (Warburg effect). This study revealed that MACC1-AS1 played a regulatory role in NOTCH1 signaling and glycolysis via PAX8 in PC, suggesting that MACC1-AS1 might serve as an novel treatment target for PC.

## Materials and methods

### Clinical samples and cell lines

The PC cell lines BxPC-3, PANC-1, MIA PaCa-2, KP-2, AsPC-1, and Capan-1 were obtained from the American Type Culture Collection (ATCC, Manassas, VA, USA). The cells were cultured following the instructions recommended by the ATCC. Two PC cohorts, composed of 98 and 124 human primary PC tissues and the paired surrounding noncancerous tissues (NCTs) were got from Ningbo First Hospital. All patients have signed informed consent, and the Clinical Research Ethics Committees of the participating institutions has approved the study. We performed the study according to the International Ethical Guidelines for Biomedical Research Involving Human Subjects (CIOMS).

### Microarray analysis

We extracted total RNA from five paired NCTs and PC tissues with RNAiso solvent (Takara, Japan), and an Agilent 2100 bioanalyzer (Agilent, CA, USA) to verify RNA integrity. Meanwhile, we performed LncRNA expression profiling via ArrayStar Human LncRNA array 2.0, and used GeneSpring GX v11.5.1 software (Agilent) to analyze data. LncRNAs were considered expressed differentially when the fold change between the PC and NCT groups > 2.0, with *P* values < 0.05.

### Quantitative RT-PCR

We applied the PrimeScript II 1st Strand Synthesis Kit (TaKaRa Biotechnology, Dalian, China) to transcribe the total RNA reversely into cDNA, and conducted qRT-PCR on the ViiA7 real-time PCR system (Applied Biosystems, Grand Island, NY, USA) with the RT-RNA PCR kit (TaKaRa). Furthermore, we normalized the relative gene expression to β-actin and used the 2^-∆∆Ct^ method to do the calculation.

### siRNA and vector construction

We synthesized the MACC1-AS1 sequence (NR_046756) via Genecopoeia (China), which was cloned into the lentiviral expression vector pWPXL and the eukaryotic expression vector (pcDNA3.1) (Invitrogen, Carlsbad, CA, USA). We obtained the siRNAs of PAX 8 and MACC1-AS1 from (GenePharma, Shanghai, China). We synthesized the verified shRNA sequence of MACC1-AS1, which was cloned into the expression lentivector as well as the pSIH-H1 shRNA cloning.

### Generation of PC cell lines with stable knockdown and overexpression of MACC1-AS1

We co-transfected the pWPXL-MACC1-AS1, pWPXL, pSIH-H1- shMACC1-AS1 or pSIH-H1 plasmid into HEK-293 T cells together with the the envelope plasmid pMD2G and packaging plasmid ps-PAX2 with Lipofectamine 2000 (Invitrogen) as being illustrated before. We gathered the virus particles 48 h post co-transfection, which were applied individually to get PC cells infected to produce stable cell lines correspondingly. Then, we performed qRT-PCR to evaluate the efficiency of MACC1-AS1 knockdown and overexpression.

### Colony formation assay and cell proliferation detection

We detected the cell activity with the Cell Counting Kit 8 (CCK-8, Dojindo, Japan) in accordance with instructions of the manufacturers. We seeded 800 to 1500 PC cells into a 6-well plate, which were kept in a medium with 10% FBS for 10 d to fulfill the colony formation assay. Then, we fixed the colonies by methanol, which were stained by 0.1% crystal violet; we used an inverted microscope to count the number of clones.

### Apoptosis analyses and cell cycle

We collected PC cells, which were fixed in 70% ethanol at ice-cold temperature. Then, we washed the fixed cells two times with PBS buffer and applied the Cell Cycle and Apoptosis Detection Kit (MultiSciences, Hangzhou, China) to perform cell-cycle analysis. We treated PC cells with 0.25 mg/mL 5-FU for 48 h to conduct cell apoptosis analysis. Next, we collected the cells and used the Annexin V-FITC/PI Apoptosis Detection Kit (RiboBio, Guangzhou, China) or Annexin V-PE/7-ADD Apoptosis Detection Kit (RiboBio) to perform apoptosis analysis.

### Cells invasion and migration tests

We performed cells invasion and migration tests with Boyden Transwell chambers (8-mm pore size, BD Biosciences) as illustrated before [10].

### In vivo tumorigenicity assay

PANC-1 (KP-2) cells stably expressing MACC1-AS1 (shMACC1-AS1) or the control vector were subcutaneously injected into either flank of the same athymic male BALB/c nude mouse (18–22 g) at 4–6 weeks of age (*n* = 6) from Shanghai Laboratory Animal Center, CAS. Four to 5 weeks post the injection, we killed the mice and detected the subcutaneous tumor growth. We killed the mice 5 weeks later and looked at the hepatic metastases. An orthotopic mouse model was used to evaluate the effect of MACC1-AS1 on hepatic metastasis. Briefly, 2 × 10^6^ KP-2 cells stably expressing MACC1-AS1 were injected into the spleen parenchyma male BALB/c nude mouse at 8 weeks of age (*n* = 5 for each group). We sacrificed the mice 6 weeks post the injection and examined hepatic metastasis. All handling procedures and animal care were conducted according to the Use of Laboratory Animals and the National Institutes of Health’s Guide for the Care. We got approval for all animal experiments from the Clinical Research Ethics Committees of Affiliated Hospital of Jiangnan University.

### RNA-seq and computational analyses

We used RNA-seq to test the mRNA expression levels of PC cells with silenced MACC1-AS1 with HiSeq3000 (Illumina, San Diego, CA, USA) at RiboBio. We applied LifeScope v2.5.1 to produce raw counts corresponding to genes that already known (a total of 20, 345 genes), align the reads to the genome, and detect the RPKM (reads per kilobase per million) values. We chose the differential genes with fold change > 1.5 and applied Gene Ontology (GO) detection for pathway enrichment by Cytoscape (ClueGo, http://www.ici.upmc.fr/cluego/cluegoDownload.shtml) with *P* < 0.01.

### RNA pull-down assays and mass spectrometry analyses

The Pierce Magnetic RNA-Protein Pull-Down Kit (Thermo Fisher, Waltham, MA, USA) was applied to perform RNA pull-down assays in accordance with the instructions of the manufacturers. Briefly, the MACC1-AS1 sequence was in vitro transcribed with biotin RNA-labeling mix and T7 RNA polymerase (Invitrogen) according to the manufacturer’s instructions. The biotinylated MACC1-AS1 RNA was incubated with streptavidin-linked magnetic beads and total cell lysates at room temperature for 2 h. The beadRNA–protein complexes were washed with 1 binding washing buffer four times. The proteins were precipitated and diluted in protein lysis buffer. Finally, we measured the retrieved proteins on Western blot analysis or SDS-PAGE gels for one-shot mass spectrometry.

### Luciferase reporter assay

The reporter construct (pGL3, Promega, Madison, WI, USA) was applied to assess the activity of NOTCH1 transcription. We transfected transiently HEK-293 T cells with the plasmids, and applied the pRL-TK Renilla luciferase plasmid as a control to modulate the variations of different wells. 36 h post the transfection, we collected the cells and used the DualLuciferase Reporter Assay System (Beyotime, Shanghai, China) to test luciferase activity.

### RNA immunoprecipitation detection

The Magna RIP RNA-Binding Protein Immunoprecipitation Kit (Millipore) was applied to perform RNA Immunoprecipitation (RIP) detection as being illustrated before. We gathered 1 × 10^7^ PC cells to be lysed by RIP lysis buffer, and co-immunoprecipitated cell extracts by the anti-PAX8 antibody (Cell Signaling Technology, Danvers, MA, USA). Meanwhile, MACC1-AS1-specific primers were used to conduct qRT-PCR analysis on the retrieved RNA. We detected the total RNA (input controls) as well as the normal mouse IgG controls simultaneously to verify that the signals being detected before were specifically from the RNAs which were bound with PAX8.

### Western blotting

We applied the PARIS Kit (Life Technologies) to separate nuclear and cytoplasmic fractions in accordance with the instructions of manufacturers. The concentration of total protein was detected with the BCA™ Protein Assay Kit (Pierce, Appleton, WI, USA). We separated the extracted proteins with SDS-PAGE, which were transferred to PVDF membranes. 5% non-fat milk was used to block the membrane, which was incubated with primary antibodies against NOTCH1 (ab65297, Abcam, Cambridge, UK, 1:800), PAX8 (ab53490, Abcam, 1:1000), Ub (sc-166,553, Santa Cruz Biotechnology, 1:500), Histone H3.1 (ab1791, Abcam, 1:500), HA (Cat#2367, Cell Signaling Technology, NY, USA, 1:2000), and anti-GAPDH (ab9484, CellSignaling, Danvers, MA, 1:1000).

### Immunohistochemistry (IHC)

PAX8 protein expression was detected with IHC analysis by PC tissue arrays, which were constructed before. We conducted IHC staining on sections of 5-mm tissue samples embedded with paraffin. In short, we incubated the slides with anti-PAX8 antibodies (cat#10336-1; ProteinTech Group, Chicago, IL, USA) overnight at 4 °C. Then, we performed the following steps with the GTVision III Detection System/Mo&Rb (Gene Tech, Shanghai, China).

### Seahorse XF analyzer respiratory assay

Cells were plated in a 24-well XF Analyzer plate (Seahorse Bioscience, North Billerica, MA, USA), the extracellular acidification rate (ECAR) and oxygen consumption rate (OCR) were measured using a Seahorse XF24 Analyzer (Seahorse Bioscience) as previously described [11].

### Statistical analysis

GraphPad Prism 7.0 software (Graph Pad Software, La Jolla, CA, USA) was applied to complete all statistical analysis. Results are shown as the mean ± SEM. The variations among different groups were compared via the x^2^ test, the Mann–Whitney U test, and Student t test. The variations of survival rates in two groups were determined with the log-rank test and Kaplan– Meier method. The independent factors that influence survival were determined by multivariate proportional hazards regression models and cox univariate. *P* values < 0.05 was deemed to be statistically significant.

## Results

### MACC1-AS1 expression was increased in PC tissues and indicates bad prognosis

LncRNA expression levels in five paired PCs and NCTs were detected to identify differentially expressed lncRNAs in PC. Compared with NCT (*P* < 0.05, fold change > 2), 427 presented dramatically differential expression with 141 downregulated genes and 286 upregulated genes in PC in the lncRNAs analyzed (Fig. 1a). The most overexpressed new lncRNA gene was MACC1-AS1, so we performed further studies with MACC1-AS1 being focused on. MACC1-AS1 upregulation in PC was verified by the expression validation in a small PC cohort. Then, we checked the expression of MACC1-AS1 in an extended PC cohort, indicating that compared to NCTs (*P* < 0.01), it was dramatically increased in PC tissues and that compared to NCTs, 63.3% (62 of 98) of the PC tissues showed upregulation of MACC1-AS1 (Fig. 1b). The expression of MACC1-AS1 was correlated positively with the stage of tumors in PC (*P* = 0.014) (Table 1). It was revealed through survival analysis that the over-expression of MACC1-AS1 was significantly involved in disease-free survival (P = 0.014, log rank = 5.603, Fig. 1c) and poor overall survival (*P* = 0.003, log rank = 7.962, Fig. 1d). Both multivariate and univariate analyses were conducted to further analyze the prognostic impact of MACC1-AS1. It was showed that the expression of MACC1-AS1 is an isolated prognostic factor for PC [*P* = 0.038; 95% confidence interval (CI), 1.017–5.043; HR, 2.216].

**Fig. 1:** The expression of MACC1-AS1 was increased in PC tissues. **a** Heatmap of dysregulated lncRNAs determined in microarray analysis via hierarchical clustering. **b** qRT-PCR was adopted to quantify the expression of MACC1-AS1 in 98 paired PC and NCTs. Compared with NCTs, MACC1-AS1 was increased in 63.3% (62 of 98) of the PC tissues. **c**-**d** Kaplan–Meier survival results of disease-free survival and overall survival based on MACC1-AS1 levels in PC samples

**Table 1:** Correlation of the expression of MACC1-AS1 in PC with clinicopathologic features

Characteristics	MACC1-AS1		P
	Low	High	
Ages (years)			
<60	32	23	0.230
≥60	17	26	
Gender			
Male	28	30	0.704
Female	21	19	
Tumor size (cm)			
<5	35	26	0.083
≥5	14	23	
Location			
Colon	25	29	0.547
Rectum	24	20	
Differentiation			
Well and moderately	40	38	0.225
Poorly	9	11	
Depth of tumor			
T1 + T2	11	9	0.632
T3	10	12	
T4	28	28	
Tumor stage			
I + II	24	13	0.014
III	20	28	
IV	5	8	

### MACC1-AS1 promoted PC proliferation and metastasis

We detected the endogenous MACC1-AS1 expression in PC cell lines, and selected KP-2/PANC-1 cells with higher/lower expression of MACC1-AS1 for the following functional tests due to their relatively high transfection efficiency and cell vitality. Colony formation and CCK-8 assays revealed that PC colony formation and cell proliferation were notably suppressed by MACC1-AS1 knockdown, whereas the overexpression of MACC1-AS1 promoted colony formation and cell proliferation (Fig. 2a-b). Furthermore, the percentage of S phase cells was reduced and cell apoptotic rate was increased with the silence of the expression of MACC1-AS1, whereas relative to control group, G1/S cell-cycle progression was promoted and PC apoptotic levels was inhibited with the aberrant expression of MACC1-AS1 (Fig. 2c–d). To avoid false positives, these experiments were also performed in BxPC-3 and AsPC-1 cell lines (Additional file 1: Figure S1). Our data showed that the same results were shown in these two cell lines. Moreover, PC carcinogenicity was suppressed under MACC1-AS1 knockdown, whereas the carcinogenicity was promoted under overexpression of MACC1-AS1 in mice (Fig. 2e). Taken together, the results indicated the promoting roles of MACC1-AS1 in the cells growth in PC. Additionally, it was revealed in Transwell assays that the invasion and migration of PANC-1 and KP-2 cells were repressed with the silencing of MACC1-AS1, which were notably promoted after overexpression of MACC1-AS1 (Fig. 2f). Besides, a mouse metastasis model of hepatic metastasis was adopted to evaluate the effect of MACC1-AS1 on in vivo metastasis. The data showed that PC hepatic metastasis was remarkably promoted with the overexpression of MACC1-AS1 (Fig. 2g).

**Fig. 2:** MACC1-AS1 promoted PC proliferation and metastasis. **a** CCK-8 outcomes of impacts of MACC1-AS1 on PC proliferation. **b** FACS analysis of impacts of MACC1-AS1 on colony formation in KP-2 and PANC-1 cells. **c**-**d** Effects of MACC1-AS1 on cell cycle and apoptosis in KP-2 and PANC-1 cells by. **e**, Nude mouse xenograft model of impact of MACC1-AS1 on carcinogenesis. **f** Representative images revealing the migration and invasion capacities of MACC1-AS1 knockdown/overexpressed PC cells. **g** Metastasis mouse model impact of MACC1-AS1 on hepatic metastasis. *P < 0.05, **P < 0.01

### MACC1-AS1 is related to PAX8

The expression of genes in MACC1-AS1–silenced KP-2 cells was detected to uncover the underlying molecular mechanism of MACC1-AS1 regarding PC. Pull-down assay was used to identify the targets which were directly regulated by MACC1-AS1. The retrieved proteins were subjected to the SDSPAGE electrophoresis analysis, and in terms of a mass spectrum analysis, we picked some additional differential bands (Fig. 3a). PAX8 was found to be a protein related to MACC1-AS1 via protein annotation, which was projected in mass spectrum analysis. The association of MACC1-AS1 and PAX8 was confirmed further in Western blotting with the retrieved proteins in the RNA pull-down assay (Fig. 3b), which was also verified in RIP assays with antibodies against PAX8 (Fig. 3c). Collectively, the outcomes showed the physical bound of MACC1-AS1 to PAX8. Several HA-tagged PAX8 deletion mutants were adopted in RIP tests to detect the exact domain of PAX8 interacting with MACC1-AS1, where the A2 domain of PAX8 is critical in terms of the interaction of PAX8 to MACC1-AS1 (Fig. 3d).

**Fig. 3:** MACC1-AS1 increased the expression and stability of PAX8. **a** SDS-PAGE was applied to analyze proteins retrieved from the pull-down assay of MACC1-AS1. **b** Pull-down assay of MACC1-AS1 with antibodies against PAX8. **c** Interaction of PAX8 with MACC1-AS1 in KP-2 cells detected by RIP assays. **d** Enrichment of FEZF1-AS1 was measured by qRT-PCR. Expression of HA-tagged pCMV-PKM2 detected by Western blot. **e** PAX8 subcellular loci in PC cells. **f** PAX8 protein expression was detected in MACC1-AS1–overexpressing PANC-1 cells by Western blot. **g** PAX8 protein levels were examined after MACC1-AS1 knockdown via Western blot. **h** Ubiquitous modification of PAX8 was suppressed by MACC1-AS1 over-expression of. *P* < 0.01

### The stability of PAX8 protein is increased by MACC1-AS1

The PAX8 subcellular localization and expression in MACC1-AS1–overexpressing or MACC1-AS1–depleted PC cells were explored to investigate the regulating role of MACC1-AS1 regarding PAX8 activity. Nevertheless, both the nuclear and total PAX8 expression profiling were dramatically down-regulated in KP-2 cells with silenced MACC1-AS1 and up-regulated in PANC-1 cells with the over-expressed MACC1-AS1 (Fig. 3e), revealing that the expression of PAX8 protein at the level of post-transcription could be increased by MACC1-AS1. In addition, the impact of MACC1-AS1 on the degradation of PAX8 was investigated in the protein synthesis inhibitor cycloheximide (CHX) to confirm the previous outcome, in which the half-life of PAX8 was prolonged with overexpression of the MACC1-AS1 in PANC-1 cells (Fig. 3f). Furthermore, we found that si-MACC1-AS1–induced endogenous PAX8 downregulation in KP-2 cells was prevented in the suppressing proteasome activity, showing that MACC1-AS1 could suppress the degradation of PAX8 through the ubiquitin-proteasome pathway (Fig. 3g). Additionally, we assessed the impact of MACC1-AS1 on ubiquitination of PAX8 in PC cells to validate the results. In conclusion, the data revealed that the expression of PAX8 is increased by MACC1-AS1 via increasing its stability and binding to it.

### MACC1-AS1 promotes tumors in PC via modulating PAX8

To explore whether MACC1-AS1 promoted tumorigenesis in PC via regulating PAX8, we investigated the impact of PAX8 on the proliferation of cells induced by MACC1-AS1. The cell growth induced by MACC1-AS1 in PC cells was blocked by the knockdown of PAX8 (Fig. 4a-b). Additionally, the increased mobility of cells in PC cells with overexpressed MACC1-AS1 was reversed with the knockdown of PAX8, and the reduced mobility of cells in PC cells with silenced MACC1-AS1 was partially recovered with the overexpression of PAX8 (Fig. 4c-d). It could be concluded here that MACC1-AS1 promotes tumorigenesis in PC via promoting the activity of PAX8.

**Fig. 4:** PAX8 regulates functions of tumor promotion of MACC1-AS1 in PC cells. **a** and **b** Increased cell livability in PC cells with over-expressed MACC1-AS1 was restored via knocking PAX8 down, but the reduction of the activity of PC cells with silenced MACC1-AS1 was abolished via the overexpression of PAX8. We detected the cell viability with CCK-8 assays. **c** and **d** MACC1-AS1–induced cell migration was partially hurdled by PAX8 knockdown, whereas the decreased cell motility in PC cells with silenced MACC1-AS1 was rescued via the overexpression of PAX8. *P* < 0.05; *P* < 0.01

### PAX8 expression level are increased in PC and correlates with the expression of MACC1-AS1 positively

The protein expression of PAX8 in 124 paired PC and NCT samples was assessed with IHC to further explore the correlation of MACC1-AS1 with PAX8 in PC tissues (Fig. 5a). It was showed in the IHC staining that relative to the paired NCTs, as many as 54% of PCs (67/124) demonstrated upregulated PAX8 expression (Fig. 5b). Meanwhile, the expression of PAX8 protein in PC tissues were related to the MACC1-AS1 expression positively (Fig. 5c, *P* < 0.001, r = 0.374), in which the positive modulation of PAX8 via MACC1-AS1 in practical PC samples was validated.

**Fig. 5:** PAX8 overexpression in PC was correlated with MACC1-AS1 positively. **a** Immunohistochemical staining of PAX8 PC tissues. **b** the expression levels of PAX8 protein were frequently up-regulated in PC tissues. **c** PAX8 expression was positively correlated with MACC1-AS1 in PC tissues (*n* = 76). **d** Kaplan–Meier survival analysis of PC patients

Overexpression of PAX8 was notably involved in lymphatic invasion (*P* = 0.015) as well as advanced carcinoma stage (*P* = 0.028). Furthermore, it was showed in the survival detection that the expression of PAX8 implies poorer prognosis in PC (Fig. 5d, *P* < 0.001, log rank = 12.7). After adjusting for gender, age, location, tumor size, TNM stage, as well as differentiation, it was indicated in multivariate analysis that the expression of PAX8 was an isolated risk factor for the survival of PC patients (*P* = 0.013; 95% CI, 1.083–4.316; HR, 2.337). Taken together, the in vivo livability of PAX8 in PC could be modulated by MACC1-AS1.

### The PAX8/NOTCH1 pathway is activated by MACC1-AS1

Luciferase assays was adopted to investigate the status of the NOTCH1 pathway in PC cells with diversed PAX8 and MACC1-AS1 expression levels to see whether NOTCH1 signaling can be activated by MACC1-AS1 via modulating the activity of nuclear PAX8. Then, in PC cells with overexpressed PAX8 or MACC1-AS1, the signaling of NOTCH1 was activated, whereas NOTCH1 activation induced by MACC1-AS1 was blocked with PAX8 with silenced expression. On the contrary, NOTCH1 activation was suppressed with MACC1-AS1 knockdown, which was restored with the overexpression of PAX8 (Fig. 6a). It was further revealed with western blot data that the phosphorylation of NOTCH1 was increased by the overexpression of MACC1-AS1, which was blocked via knocking PAX8 down (Fig. 6b). In contrast, NOTCH1 phosphorylation was suppressed via knocking MACC1-AS1 down, which was restored with PAX8 overexpression. Meanwhile, the overexpression of MACC1-AS1–PC cells also dramatically increased downstream targets of the NOTCH1 pathway (BIRC5, SNAIL1, SLUG, CCND1, MMP2, CDH1, as well as MMP9), and PAX8 knockdown could partially suppress their expression, which was consistent with the outcomes above (Fig. 6c). Taken together, the results showed that the NOTCH1 pathway is activated by MACC1-AS1 through PAX8.

**Fig. 6:** MACC1-AS1 activated NOTCH1 signaling and promoted glycolysis by PAX8. **a** the NOTCH1 pathway was activated by MACC1-AS1 via PAX8. **b** MACC1-AS1 induced NOTCH1 phosphorylation in PC cells via PAX8. **c** downstream elements of the NOTCH1 pathway were activated by MACC1-AS1 via PAX8. **d**-**e** the lactate production and pyruvate kinase activity were facilitated by MACC1-AS1 via modulating PAX8 in the KP-2 cell. **f**-**g** ECAR and OCR were promoted by MACC1-AS1 via modulating PAX8 in the KP-2 cell. *P* < 0.05, *P* < 0.01

### MACC1-AS1 prompts aerobic glycolysis via PAX8

Next, we determined whether the pyruvate kinase activity of PAX8 is affected by MACC1-AS1. It was found that the lactate production and pyruvate kinase activity were increased with the overexpression of MACC1-AS1, whereas they were notably hurdled with the knockdown of PAX8 in PC cells (Fig. 6d-e). Nevertheless, the lactate production and pyruvate kinase activity in PC cells were suppressed with the knockdown of MACC1-AS1, but they were restored with the overexpression of PAX8. Moreover, the OCR and ECAR in PC cells were inhibited by MACC1-AS1 knockdown, but were restored by PAX8 overexpression (Fig. 6f-g). It could be concluded here that together with its main modulatory impact on the protein kinase activity of PAX8, MACC1-AS1 might facilitate aerobic glycolysis via increasing the pyruvate kinase activity of PAX8 (Fig. 7).

**Fig. 7:** Schema presented the mechanism through which NOTCH1 aerobic glycolysis and signaling in PC cells were modulated by MACC1-AS1

## Discussion

Gene expression can be regulated by LncRNAs in multiple ways, such as transcriptional and posttranscriptional processing, as well as chromatin modification [12]. There have been reports on the extensive modulatory roles of lncRNA in carcinogenesis and the progression [13]. Previously reports detected several lncRNAs expressed differentially in PC, such as UCA1, DUXAP8, Linc00511, and Linc01060, which have been determined to be underlying oncogenes [14–16]. MACC1-AS1, a highly overexpressed lncRNA and a novel detected carcinogenic lncRNA in gastric cancer [17, 18]. Nevertheless, the molecular mechanisms and potential function of MACC1-AS1 in PC is still unclear.

In our study, we uncovered that the expression of MACC1-AS1 was increased in PC tissues, and projected poorer prognosis, which was in compliance with the reports issued before. It was showed in functional trials that MACC1-AS1 PC carcinogenesis and metastasis were dramatically facilitated both in vivo in and vitro. Furthermore, we observed that the apoptosis of PC cells is suppressed by MACC1-AS1. MACC1-AS1 is the cognate antisense lncRNA of MACC1. MACC1 is a highly conserved transcriptional inhibitor modulating the development of nervous system, which is a promising target for cancer therapy [17]. Zhao et al. has found that the MACC1-AS1/MACC1 axis exerts as a regulator of metabolic plasticity via enhacing antioxidant and glycolysis production [18]. Generally, the function of MACC1 in human carcinomas is still not clear.

NOTCHs, especially NOTCH1, are well known for their modulatory impacts on cell proliferation, metastasis, and apoptosis in human carcinomas. PAX8, a modulator of the signaling of NOTCH1 in PC, was determined to be a critical downstream target of MACC1-AS1 via screening and verification in experiments. PAX8 could play a role as a protein kinase in the nucleus, which modulate various genes and pathways related to cancer, such as BNC2, HOXB4, SP6 as well as WNT4 [19]. Our study shows that cytoplasmic PAX8 was slightly increased in PC cells with overexpressed MACC1-AS1, resulting in promoted aerobic glycolysis, indicating that PC carcinogenesis and development were facilitated by MACC1-AS1 via modulating activities of both pyruvate kinase and protein kinase of PAX8. Whether or how MACC1-AS1 regulates the sub-cellular site of PAX8 is still unclear, which requires additional investigations to determine whether there is “cross-talk” between these modulatory mechanisms.

## Conclusions

It can be concluded that our study shows that MACC1-AS1 is upregulated in PC, which is involved in poorer survival. The proliferation and metastasis of PC cells were increased by MACC1-AS1 via regulating glycolysis and PAX8/NOTCH1 signaling, suggesting the first evidence of a MACC1-AS1/PAX8 network in PC. The outcomes demonstrate that MACC1-AS1/PAX8 signaling could serve as an optimal treatment target in PC.

## Additional file

Additional file 1: MACC1-AS1 promoted the proliferation and metastasis in BxPC-3 and AsPC-1 cell lines. (TIF 2123 kb)

## Data Availability

The authors declare that the data supporting the findings of this study are available within the article.

## Abbreviations

ATCC: American Type Culture Collection
GO: Gene ontology
IHC: Immunohistochemistry
lncRNAs: Long ncRNAs
NCTs: Noncancerous tissues
PC: Pancreatic carcinoma
RIP: Perform RNA Immunoprecipitation
